# Evaluating Histological Subtypes Classification of Primary Lung Cancers on Unenhanced Computed Tomography Based on Random Forest Model

**DOI:** 10.1155/2023/8964676

**Published:** 2023-02-06

**Authors:** Jianfeng Huang, Wei He, Haijia Xu, Shan Yang, Jiajun Dai, Weifeng Guo, Mengsu Zeng

**Affiliations:** ^1^Department of Radiology, Zhongshan Hospital, Fudan University, Shanghai 200032, China; ^2^Department of Vascular Surgery, Zhongshan Hospital, Fudan University, Shanghai 200032, China; ^3^School of Basic Medical Sciences, Fudan University, Shanghai 200032, China

## Abstract

Lung cancer is the leading cause of cancer-related death in many countries, and an accurate histopathological diagnosis is of great importance in subsequent treatment. The aim of this study was to establish the random forest (RF) model based on radiomic features to automatically classify and predict lung adenocarcinoma (ADC), lung squamous cell carcinoma (SCC), and small cell lung cancer (SCLC) on unenhanced computed tomography (CT) images. Eight hundred and fifty-two patients (mean age: 61.4, range: 29–87, male/female: 536/316) with preoperative unenhanced CT and postoperative histopathologically confirmed primary lung cancers, including 525 patients with ADC, 161 patients with SCC, and 166 patients with SCLC, were included in this retrospective study. Radiomic features were extracted, selected, and then used to establish the RF classification model to analyse and classify primary lung cancers into three subtypes, including ADC, SCC, and SCLC according to histopathological results. The training (446 ADC, 137 SCC, and 141 SCLC) and testing cohorts (79 ADC, 24 SCC, and 25 SCLC) accounted for 85% and 15% of the whole datasets, respectively. The prediction performance of the RF classification model was evaluated by F1 scores and the receiver operating characteristic (ROC) curve. On the testing cohort, the areas under the ROC curve (AUC) of the RF model in classifying ADC, SCC, and SCLC were 0.74, 0.77, and 0.88, respectively. The F1 scores achieved 0.80, 0.40, and 0.73 in ADC, SCC, and SCLC, respectively, and the weighted average F1 score was 0.71. In addition, for the RF classification model, the precisions were 0.72, 0.64, and 0.70; the recalls were 0.86, 0.29, and 0.76; and the specificities were 0.55, 0.96, and 0.92 in ADC, SCC, and SCLC. The primary lung cancers were feasibly and effectively classified into ADC, SCC, and SCLC based on the combination of RF classification model and radiomic features, which has the potential for noninvasive predicting histological subtypes of primary lung cancers.

## 1. Introduction

Random forest (RF) algorithm, proposed by Leo Breiman [1], is an ensemble learning algorithm based on classification and regression trees (CART). The RF algorithm contains several CARTs, and each one is independent. Therefore, the RF algorithm performs insensitively to the overfitting problem of the training cohort and has superior noise immunity, which is not sensitive to default values [2]. The RF algorithm is widely applied in various fields, such as life sciences because RF classification models are versatile, have high prediction accuracy, and provide additional information such as variable importance [3]. According to literature reports, RF algorithms have excellent performance in evaluating the progression, prognosis, and gene mutation expression of various diseases [4–10].

Lung cancer is the leading cause of cancer-related death in many countries, and the accurate histopathological diagnosis is of great importance in subsequent treatment [11, 12]. In previous studies, the RF model was mostly applied to detecting lung cancer, the classification of benign and malignant pulmonary nodules, and the analysis of lung cancer prognosis [13–16]. However, for therapeutic purposes, primary lung cancers fall into three major subtypes: lung adenocarcinoma (ADC), lung squamous cell carcinoma (SCC), and small cell lung cancer (SCLC), and distinguishing among subtypes is still particularly challenging. In this study, our aim is to establish a classification model combining the RF algorithm and radiomic features of unenhanced CT images to classify the primary lung cancers into ADC, SCC, and SCLC and to evaluate the prediction performance.

## 2. Materials and Methods

### 2.1. Study Population

Nine hundred and twenty patients with histopathologically confirmed primary lung cancer from January 2013 to August 2018 at Zhongshan Hospital, Fudan University, were retrospectively studied. The inclusion criteria were: (1) diagnosis of ADC, SCC, or SCLC confirmed by puncture or surgical specimen; (2) preoperative CT examination within 2 weeks before surgery. The exclusion criteria were: (1) patients receiving other treatments such as chemotherapy and radiotherapy before surgery; (2) patients with lesion boundaries that were difficult to identify on CT images; (3) patients with inadequate quality images on CT; (4) patients with two or more histopathological subtypes of primary lung cancer; and (5) patients with the lesion less than 1 cm in diameter, avoiding partial volume effects. Eight hundred and fifty-two patients with primary lung cancer (525 ADC, 161 SCC, and 148 SCLC) were ultimately included in this study. All study procedures were approved by the Ethics Committee of Zhongshan Hospital, Fudan University.

### 2.2. Protocol of Unenhanced Computed Tomography and Segmentation

All patients had preoperative CT examinations performed within 2 weeks before the puncture or surgery under breath-hold conditions at the end of inspiration, from the thoracic inlet to the diaphragm, by experienced radiologists. The parameters of *μ*CT 760 (Shanghai United Imaging Healthcare) were: tube voltage = 120 kV, tube current = 130 mA, slice thickness = 1 mm, and the parameters of LightSpeed 16 (GE Healthcare) were: tube voltage = 120∼140 kV, tube current = 140 mA, and slice thickness = 1 mm. All image data were stored in DICOM format.

ITK-Snap software (version 3.6.0) was used to segment each layer of the tumor lesions on the CT images in all cases to obtain a three-dimensional region of interest (ROI) [17], which was output in mha format for analysis (see Figure 1). The histopathological results (ADC, SCC, or SCLC) of each case were matched to the segmentation results. All procedures of ROI segmentation were performed by two experienced radiologists and finally confirmed by a senior radiologist.

## 3. Establishment of Random Forest Classification Model

### 3.1. Extraction of Radiomic Features

PyRadiomics package implemented in Python was used to extract radiomic features [18] (see Figure 2). The radiomic features of both the original and wavelet denoised (db2 was set as the wavelet basis) images were extracted, such as shape-based features, firstorder statistics, the gray level co-occurrence matrix (GLCM), the gray level run length matrix (GLRLM), the neighboring gray tone difference matrix (NGTDM), the gray level dependence matrix (GLDM), and the gray level size zone matrix (GLSZM) (see Figure 2).

The features were first normalized to the range 0– 1, and then the support vector machine (SVM) was used to filter the features (see Figure 2). The variance inflation factor (VIF) was used to detect the collinearity of features which made the area under the receiver operating characteristic (ROC) curve (AUC) of SVM classification greater than 0.5, and features with VIF less than or equal to 5 were selected (see Figures 2 and 3). The formula of VIF is given as follows:

(1) $$\begin{array}{c} VIF=\frac{1}{1-R^{2}}\text{.} \end{array}$$

The spatially uniform relevant features (ReliefF) algorithm was used to further filter the features (see Figure 2), and the final retained radiomic features were summarized in Table 1 (see Table 1). The importance score of each feature for predicting the histopathological subtypes of primary lung cancer are shown in Figure 4 (see Figure 4).

### 3.2. Random Forest Algorithm

Selected radiomic features were used to establish and RF classification model with the following parameters: “n_estimators” = 100; “max_depth” = 11; “min_samples_split” = 2; and “min_samples_leaf” = 4. In this study, 85% of the whole data (724 in all, 446 ADC, 137 SCC, and 141 SCLC, respectively) were randomly divided into the training cohort which was used for feature selection as well as model fitting, and 5-fold cross-validation was used to validate in the training cohort, while the remaining 15% (128 in all, 79 ADC, 24 SCC, and 25 SCLC, respectively) were divided into the testing cohort for validation (see Table 2 and Figure 5).

### 3.3. Statistical Analysis

Statistical analysis was performed using SPSS software (Version 22.0) and Python 3.8.0 (NumPy packages). Categorical variables were presented as quantities (percentages) and compared using the chi-square test or Fisher's exact test, while continuous variables were presented as the mean ± SD if normally distributed, and compared using the Kruskal–Wallis H test because of the heterogeneity of variance. AUC, sensitivity, specificity, and accuracy were used to evaluate the predictive performance of the classification model. In addition, the F1 score was also used to evaluate the efficiency of the classification models. A two-tailed *p* value <0.05 was considered statistically significant.

## 4. Results

### 4.1. Patients' Clinical Characteristics

Patients' clinical baselines and characteristics were summarized in Table 3 (see Table 3). Eight hundred and fifty-two patients with primary lung cancer (mean age: 61.4, range: 29–87, male/female: 536/316) were ultimately included in this study, including 525 patients with ADC (61.6%, mean age: 60.4, range 29–87, male/female: 247/278), 161 patients with SCC (18.9%, mean age: 64.0, range 34–82, male/female: 148/13), and 166 patients with SCLC (19.5%, mean age: 62.1, range 38–82, male/female: 141/25), respectively, and randomly divided into the training cohort (724 patients) and testing cohort (128 patients) in the ratio of 85% to 15% (see Table 2). Notably, the differences in age, gender, and TMN stage of patients among the three subtypes were statistically significant.

### 4.2. Predictive Performance of Random Forest Classification Model

Twenty radiomic features were ultimately selected after features were extracted and filtered from the unenhanced CT to establish the RF classification model, including 7 firstorder features, 3 GLSZM features, 2 GLRLM features, 4 GLDM features, and 4 NGTDM features.

For the RF classification model, ROC-AUC was 0.74, 0.77, and 0.88 for the ADC, SCC, and SCLC, respectively, on the testing cohort. The average AUC for the three subtypes of classification was 0.80 (95% CI = 0.769–0.813) (see Figure 6). In addition, the F1 scores achieved 0.80, 0.40, and 0.73 in ADC, SCC, and SCLC, respectively, and the weighted average F1 score was 0.71. Notably, the precisions were 0.72, 0.64, and 0.70, the recalls were 0.86, 0.29, and 0.76 and the specificities were 0.55, 0.96, and 0.92 in ADC, SCC, and SCLC (see Table 4).

## 5. Discussion

The histopathological diagnosis and classification of primary lung cancers are of great importance and crucial clinical value for the decision of optimal and individualized treatment schedules and the evaluation of prognosis [19]. In this study, RF algorithms combined with radiomic features on unenhanced CT images were used for noninvasive and preoperative prediction of subtype's classification of primary lung cancer. Radiomic features were extracted and filtered from enhanced CT images, and the ultimately 20 selected features were used to establish the RF classification model, which was trained and validated using the training cohort and the testing cohort. To be noted, 5-fold cross-validation was used for more accurate precision. Finally, the prediction performance of the model in classifying the three major subtypes (ADC, SCC, and SCLC) of primary lung cancers was evaluated.

The results showed that the RF classification model was able to accurately classify the three subtypes on the testing cohort (AUC = 0.80). Particularly, the model performed better in predicting SCLC (AUC = 0.88) than ADC (AUC = 0.74) and SCC (AUC = 0.77). However, this model tended to misclassify SCC as ADC, thus the recalls of the RF model in ADC (0.86) and SCLC (0.76) were excellent, while inferior in SCC (0.29). It was probably because (1) the sample of SCC (161) was limited and much fewer than that of ADC (525) and (2) most of the SCC included in this study were central-type lung cancer, which was difficult to distinguish on the CT images, leading to inaccurate segmentation of ROI. Certainly, the reason for the misclassification deserved further investigation and verification. In this study, the selected 20 radiomic features were not the same as the features in previous studies (com_radNet model), but they improved the predictive classification of SCLC [20].

Previously, a large number of studies have proven the excellent performance of the RF algorithm in classifying benign and malignant pulmonary nodules on CT and PET/CT [21–24]. Zhu et al. classified ADC and SCC in 129 patients with non-SCLC (NSCLC) based on 5 radiomic features with an AUC, specificity, and sensitivity of 0.89, 0.90, and 0.83, respectively, on the validation cohort [25]. Liu et al. classified 349 patients with NSCLC, including not only ADC and SCC but also large cell carcinoma and not otherwise specified based on radiomic features combined with SVM, and the classification accuracy was 0.86 on the testing set [26]. In this study, we expanded the samples and also investigated the classification between SCLC and NSCLC, with the considerably improved predictive performance of the RF classification model. To our knowledge, the only radiomics-based study on the classification of SCLC and NSCL identified ADC, SCC, and SCLC in a two-by-two comparison. The results showed good classification performance between ADC and SCLC (AUC = 0.86) and between ADC and SCC (AUC = 0.80) on unenhanced CT images and better performance on enhanced CT, but neither could effectively classify SCC and SCLC (AUC = 0.62 and 0.66). To note, the RF classification model was able to classify SCLC with great performance in our study.

The study has some limitations. First, the sample of ADC was much larger than that of SCC and SCLC, mainly due to the different morbidities, which may affect the diagnostic performance of the model [27]. Furthermore, although we have excluded cases with blurred tumor borders, the possibility of missegmentation of nontumor tissues existed. Finally, large multicenter, prospective studies are essential for model expansion and optimization.

## 6. Conclusions

In conclusion, the noninvasive histopathological subtype classification of primary lung cancers has great clinical significance and value. In our study, the primary lung cancers were feasibly and effectively classified into ADC, SCC, and SCLC based on the combination of the RF classification model and radiomic features. Large studies are needed to optimize and validate the performance of the model. The RF classification model combined with radiomic features on unenhanced CT images is able to provide additional information about patients and has the potential for clinical applications.

## Figures and Tables

**Figure 1:** Segmentation of lesions on CT images and 3D ROI for (a) adenocarcinoma, (b) squamous cell carcinoma, and (c) small cell lung cancer.

**Figure 2:** The flowchart for extraction and selection radiomic feature.

**Figure 3:** Correlation between radiomic features. 0 represents no correlation.

**Figure 4:** The importance score of each feature for predicting the histopathological subtypes of primary lung cancer.

**Figure 5:** Flowchart of random forest algorithm.

**Figure 6:** ROC curve analysis of the RF classification model. The black solid line represents SCLC (class 0), the blue solid line represents ADC (class 1), the green solid line represents SCC (class 2), and the dark blue dotted line represents the average.

**Table 1:** Selected radiomic features.

No	Radiomics features
0	wavelet2-LLL_firstorder_RootMeanSquared
1	wavelet-HHH_ngtdm_Contrast
2	original_firstorder_InterquartileRange
3	wavelet2-HHH_glszm_SmallAreaLowGrayLevelEmphasis
4	wavelet2-HLH_firstorder_Mean
5	wavelet2-LHL_firstorder_Kurtosis
6	original_gldm_LargeDependenceHighGrayLevelEmphasis
7	wavelet2-LHH_glszm_SmallAreaLowGrayLevelEmphasis
8	wavelet-LHL_ngtdm_Complexity
9	original_glszm_GrayLevelNonUniformity
10	wavelet-LLH_firstorder_Kurtosis
11	original_ngtdm_Strength
12	wavelet-HLH_gldm_LargeDependenceHighGrayLevelEmphasis
13	wavelet2-HHH_glrlm_GrayLevelVariance
14	original_glrlm_RunVariance
15	wavelet2-LLH_gldm_LargeDependenceHighGrayLevelEmphasis
16	original_gldm_LowGrayLevelEmphasis
17	wavelet2-LLH_ngtdm_Strength
18	wavelet-LHH_firstorder_Kurtosis
19	original_firstorder_Kurtosis

**Table 2:** Cases in the training and testing cohort.

	Training (*n* = 724, 85%)	Testing (*n* = 128, 15%)
ADC	446	79
SCC	137	24
SCLC	141	25

**Table 3:** Demographics and characteristics.

	ADC (*n* = 525)	SCC (*n* = 161)	SCLC (*n* = 166)	*p* values
Gender				<0.05
Male	247 (47.0%)	148 (91.9%)	141 (84.9%)	
Female	278 (53.0%)	13 (8.1%)	25 (15.1%)	

Age				<0.05
Mean ± SD	60.4 ± 10.5	64.0 ± 8.1	62.1 ± 9.5	
Range	18–87	23–82	41–86	

TNM				<0.05
I	139 (26.5%)	56 (34.8%)	12 (7.2%)	
II	70 (13.3%)	41 (25.5%)	19 (11.4%)	
III	91 (13.3%)	47 (29.2%)	57 (34.3%)	
IV	225 (42.9%)	17 (10.6%)	78 (47.0%)	

**Table 4:** Prediction performance of the RF classification model.

Subtypes	F1 score	Precision	Recall	Specificity
ADC	0.80	0.76	0.86	0.55
SCC	0.40	0.64	0.29	0.96
SCLC	0.73	0.70	0.76	0.92

## Data Availability

The datasets used and/or analysed during the current study are available from the corresponding author upon request.
